# Notch-1 Signaling Promotes the Malignant Features of Human Breast Cancer through NF-κB Activation

This article has been retracted.

**DOI:** 10.1371/journal.pone.0095912

**Published:** 2014-04-23

**Authors:** Li Li, Fenglong Zhao, Juan Lu, Tingting Li, Hong Yang, Chunhui Wu, Yiyao Liu

**Affiliations:** Department of Biophysics, School of Life Science and Technology, University of Electronic Science and Technology of China, Chengdu, Sichuan, P.R. China; Case Western Reserve University, United States of America

## Abstract

The aberrant activation of Notch-1 signaling pathway has been proven to be associated with the development and progression of cancers. However, the specific roles and the underlying mechanisms of Notch-1 signaling pathway on the malignant behaviors of breast cancer are poorly understood. In this study, using multiple cellular and molecular approaches, we demonstrated that activation of Notch-1 signaling pathway promoted the malignant behaviors of MDA-MB-231 cells such as increased cell proliferation, colony formation, adhesion, migration, and invasion, and inhibited apoptosis; whereas deactivation of this signaling pathway led to the reversal of the aforementioned malignant cellular behaviors. Furthermore, we found that activation of Notch-1 signaling pathway triggered the activation of NF-κB signaling pathway and up-regulated the expression of NF-κB target genes including MMP-2/-9, VEGF, Survivin, Bcl-xL, and Cyclin D1. These results suggest that Notch-1 signaling pathway play important roles in promoting the malignant phenotype of breast cancer, which may be mediated partly through the activation of NF-κB signaling pathway. Our results further suggest that targeting Notch-1 signaling pathway may become a newer approach to halt the progression of breast cancer.

## Introduction

Breast cancer is the most commonly diagnosed malignant tumor in women of all races and is the second leading causes of cancer death in women of most races. Breast cancer is commonly treated by a combination of surgery, chemotherapy, radiotherapy, and hormone therapy. With screening and continuous development of new adjuvant therapies, current 5-year survival rates are nearly 90%. Despite the improvements, the long term recurrent rates can be as high as 20%, and metastasis at diagnosis and metastatic relapse after the initial treatment remain an incurable disease and the main cause of death of breast cancer [1], [2]. Understanding the molecular mechanisms underlying the malignant behaviors of breast cancer cells would provide lead molecules for targeted therapy [3].

Notch signaling pathway is an evolutionarily conserved signaling pathway that has been shown to regulate many cellular processes including cell proliferation, differentiation, apoptosis, and survival [4]–[6]. In mammalian cells, Notch signaling pathways include four transmembrane receptors (Notch-1 to 4) and five ligands (Delta-like 1, 3, 4, Jagged 1, 2). Notch receptor is a single-pass transmembrane protein consisting of extracellular, transmembrane and intracellular domains [7]. Notch signaling is activated by ligand-receptor binding between the neighboring cells. Once activated, Notch-1 is cleaved by γ-secretase and releases the Notch-1 intracellular domain (NICD) from the plasma membrane, which then translocates into the nucleus to engage other transcription factors and regulate the expression of target genes including some members of Hes and Hey gene families. The Notch signaling pathway regulates the normal development of many tissues and cell types through its cellular context-dependent effects on cell lineage specification, cell proliferation, differentiation, and apoptosis [8]–[10]. Dysregulated Notch signaling has been reported in many tumors [8], [11], [12] including cervical cancer [13], pancreatic cancer [14], squamous cell carcinoma of the head and neck [15], renal carcinoma [16], B- and T-cell–derived tumor cells of Hodgkin, anaplastic large cell lymphoma [17], and invasive human pancreatic cancer [18]. In breast cancer, increased expression of Notch-1 and Jagged-1 has been reported to be correlated with dramatic reduction of overall survival [2]. Knockdown of Notch-1 generated therapeutic effects on estrogen receptor α–negative breast cancers [19]. All these reports clearly suggested a potential link between Notch-1 signaling and the development of human breast cancer.

NF-κB is a transcription factor that plays an important role in innate immunity and is a master regulator of inflammation. At resting conditions, NF-κB complex is sequestered in cytoplasm through binding to the inhibitor of NF-κB (IκB). Upon activation, IκB is phosphorylated and destined for ubiquitin-mediated proteosome degradation. The free NF-κB complex then translocates to the nucleus and induces the expression of its downstream target genes [20], [21]. Other than its roles in innate immunity and inflammation activation of NF-κB signaling was shown to regulate a wide variety of cellular processes including cell proliferation, differentiation, and apoptosis. Moreover, it has been reported that activation of NF-κB signaling pathway also might contribute to tumor initiation and progression (migratory and invasive phenotype) [22]–[24]. The latter is most likely associated with increased expression of matrix metalloproteinases (MMPs) and endothelial growth factor (VEGF) which facilitates distal metastases [25], [26] and tumor-associated microvascular invasion [4], [27], respectively.

However, it is still unknown how the cross-talk between Notch-1 and NF-κB signaling pathways regulates the malignant behaviors of human breast cancer. In this report, we provided evidences that activation of the Notch-1 signaling pathway (1) promoted the malignant phenotype of human breast cancer line, MDA-MB-231 cells, (2) activated NF-κB signaling pathway, and (3) up-regulated the expression of NF-κB target genes including MMP-2/-9 and VEGF that are known to facilitate tumor invasion and metastasis. Our findings suggest that activation of Notch-1 signaling pathway promotes the malignant phenotype of human breast cancer via NF-κB. Notch-1 signaling pathway is possibly a new target for the treatment of breast cancer.

## Materials and Methods

### Reagents and chemicals

Cell culture medium L15, penicillin and streptomycin were purchased from Gibco (Grand Island, NY, USA). Bradford protein assay kit, cell counting kit (CCK-8), rabbit anti-human p65 polyclonal antibody, Cy3-labeled goat anti-rabbit secondary polyclonal antibody, 4′,6-diamidino-2-phenylindole dihydrochloride (DAPI), nuclear and cytoplasmic protein extraction kit, and biotin-labeled NF-κB oligonucleotides were obtained from Beyotime Institute of Biotechnology (Jiangsu, China). Fetal bovine serum (FBS) was from HyClone (Logan, Utah, USA). Matrigel and Annexin V-cy5 were purchased from BD Biosciences (CA, USA). Trizol and Calcein-AM were from Invitrogen (Carlsbad, CA, USA), and Transwell cell culture inserts were from Millipore (MA, USA). All other chemicals were from Sigma-Aldrich (St. Louis, MO, USA) unless specified otherwise.

### Cell culture

Human breast cancer cell line, MDA-MB-231, was obtained from American Type Culture Collection (ATCC, Manassas, VA, USA). Cells were maintained and propagated in L15 culture medium supplemented with 10% FBS, 100 mg/ml streptomycin and 100 units/ml penicillin at 37°C in a humidified incubator containing 5% CO_2_.

### Plasmid construction and transient transfection of MDA-MB-231 cells

cDNA encoding Notch-1 intracellular domain (NICD) was obtained by reverse transcription-polymerase chain reaction (RT-PCR) using RNA from U251 cells. The cDNA was further amplified by PCR with sense primer (5′-SEQUENCE-3′) containing a BamHI restriction site and anti-sense primer (5′-SEQUENCE-3′) containing a HindIII restriction site. The PCR products were purified and then cloned into pcDNA3.1(+). The identify of plasmid was confirmed by DNA sequencing, which was designated as pcDNA3.1(+)-NICD. Oligonucleotides containing shRNA candidate for Notch-1 (5′-CAGTTGTGCTCCTGAAGAA-3′) or scramble shRNA (5′-CGCTGAGTACTTCGAAATGTC-3′) were cloned into the psi-U6 respectively. The identities of them were confirmed by DNA sequencing.

Twenty-four hours prior to transfection, MDA-MB-231 cells seeded at 2×10^5^/well in a 6-well plate. Cells were transfected with Lipofectamine LTX (Invitrogen) according to manufacturer's protocols. Briefly, 11.25 µl Lipofectamine LTX and 2.5 µg plasmids of NICD, Notch-1 shRNA or scramble shRNA were diluted in 100 µl Opti-MEM (Invitrogen), and then incubated for 30 min at room temperature. Following complex formation, the plasmids/Lipofectamine LTX complexes were added dropwise to the cells and mixed gently. The cells were continued to incubate for 48 hours for further downstream analysis.

### Cell proliferation assay

The transfected MDA-MB-231 cells were trypsinized and seeded at a density of 1×10^4^ cells/well onto the 96-well plate and cultured for 24 or 48 hours. At each time point, cell proliferation was evaluated using CCK-8 assay kit (Beyotime, Jiangsu, China) according to the manufacturer's instructions. Briefly, 10 µl of the cell counting kit solution was added to each well and incubated for 1 hour at room temperature. The absorbance values of all the samples were recorded by a microplate reader (Model 680, Bio-Rad, PA, USA) at the wavelength of 450 nm.

### Colony formation assay

The anchorage dependent growth of tumor cells was investigated by monolayer colony formation assay as described previously [28]. The transfected MDA-MB-231 cells were trypsinized 48 hours after transient transfection, 4,000 cells were added to 35-mm dishes containing 2 ml 10% complete medium and cultured for 8 days for colony formation. The colonies were stained with 1% crystal violet after methanol fixation, washed extensively to remove excess dye and imaged using a camera. Quantification of colony formation was performed by adding 0.5 ml 10% acetic acid to each plate with the absorbance evaluated at 450 nm. The experiments were performed in triplicate.

### Soft agar assay

Anchorage-independent growth of tumor cells was performed in 24-well plate as described previously [29], [30]. After solidation of the lower layer of 1% agarose, 4×10^3^ transfected MDA-MB-231 cells resuspended in serum-free L15 media containing 0.3% agarose (maintained at 40°C water bath) were overlaid onto the lower layer and to allow solidify. Then 400 µl of growth media was added on the top of the second layer. The cells were incubated at 37°C for 24 days until visible colonies were formed. The colonies were counted through microscopy and photographed. The experiments were performed in triplicate.

### Cell cycle assay

MDA-MB-231 cells (3×10^5^ cells) were seeded into each well of a six-well plate. After 24 hours, the cells were transfected with NICD, shRNA or empty vector. Transfected cells were harvested at 48 hours after transfection, washed twice with ice-cold PBS and resuspended in 1 ml of PBS. Cells were fixed with 70% ethanol before stained with propidium iodide (PI). DNA content was determined by FACScan flow cytometer (BD Biosciences) and cell cycle analysis was analyzed using the ModFit software (Verity) [31].

### Cell apoptosis assay

For Calcein-AM and PI co-staining, cells after various aforementioned treatments were washed with PBS and stained by a mixture of calcein-AM and PI solution for 20 min. Fluorescence images of cells were then recorded using an inverted fluorescent microscope (Nikon TE-2000U, Japan).

Annexin V/PI double-staining was performed as previously described [32]. The transfected MDA-MB-231cells were harvested by trypsinization, and stained with Annexin V-cy5 and PI in Annexin V binding buffer for 15 min at room temperature in the dark according to the manufacturer's instructions (BD Pharmingen). The data were analyzed using FlowJo software (Tree Star Inc., Ashland, USA).

### Cell adhesion assay

Transfected MDA-MB-231 cells were seeded at 3,000 cells/well in 96-well plates pre-coated with Matrigel (BD Biosciences). Cells were allowed to adhere for one hour. After washing three times with PBS, adherent cells were stained with crystal violet after fixation with methyl alcohol for 30 min. At least five random fields from each group were photographed and the numbers of adherent cells were counted.

### Cell invasion assay

Cell invasion assay was performed as described previously [33], [34] with some modifications. Briefly, 1×10^5^ transfected cells in 200 µl serum-free media were plated onto the top chamber that had been previously coated on the bottom surface with Matrigel (3.4 µg/mL, BD Biosciences) and inserted into the lower chamber containing 600 µl of 10% complete media. After 24-hour incubation, cells remaining on the top of the transwell were removed by swiping with a damp cotton swab and those migrating to the bottom of the transwell were stained with crystal violet, mounted on glass coverslips, imaged with an inverted microscopy (Nikon TE-2000U, Japan), and quantified by averaging five different fields. The experiment was repeated three times.

### Monolayer wound healing assay

The cells were transiently transfected with plasmids encoding NICD, Notch-1 shRNA, or scramble shRNA as described above. After 24-hour incubation, the monolayer was scratched with a pipette tip, washed with PBS to remove floating cells and refreshed with serum-free media. The same fields were photographed on day 0 (0 hour), day 1 (24 hours), and 2 (48 hours) under an inverted fluorescence microscope (TE-2000U, Nikon, Japan). Wound area was measured by ImageJ software and plotted as percentage of wound closure relative to day 0. More than five random fields were selected and mean value per field was expressed.

### RNA extraction and quantitative real time-PCR

Total RNA was prepared from MDA-MB-231 cells using the Trizol (Invitrogen) according to the manufacturer's instructions. One microgram of total RNA of each sample was used for reverse transcription using the Superscript II reverse transcriptase (Invitrogen) in a 20 µl reaction volume. All quantitative PCR were performed using SYBR *Premix Ex Taq* II system (Tli RNaseH Plus) (Takara), and the amplification thresold (Ct) of each gene was normalized to that of β-actin. The comparative Ct method was used to calculate fold changes. Efficiency for all primer pairs were 95–100%. Primer pairs used were Notch-1 (forward, 5′-AACAGCGAGGAAGAGGAGGA-3′; reverse, 5′-GC ATCAGAGCGTGAGT AGCG-3′), Bcl-xL (forward, 5′-AAAAGATCTTCCGGGGG CTG-3′; reverse, 5′-CCCGGTTGCTCTGAGACATT-3′), cyclin D1 (forward, 5′-AA AAGATCTTCCGGGGGCTG-3′; reverse, 5′-CCCGGTTGCTCTGA GACATT-3′), Hes-1 (forward, 5′-AAAAGATCTTCCGGGGGCTG-3′; reverse, 5′-CCCGGTTGCT CTAGACATT-3′), Survivin (forward, 5′-TTCTCAAGGACCACCGCATC-3′; reverse, 5′-AATGGGGTCGTCATCTGGCT-3′), VEGF (forward, 5′- TTCTCAAG GACCACCGCATC-3′; reverse, 5′-AATGGGGTCGTCAT CTGG T-3′), and β-actin (forward, 5′-AGTTGCGTTACACCCTTTCTTG-3′; reverse 5′-TCACCTTCACCG TTCCAGT TT-3′).

### Gelatin zymography

Non-transfected and transfected MDA-MB-231 cells were cultured in serum-free media for 48 hours. The conditioned media was collected and concentrated by lyophilization, which were then re-dissolved into 0.5 ml of Milli-Q water. The protein concentration was quantified with Bradford protein assay (Beyotime, Jiangsu, China). Ten µg of each reconstituted conditioned media were resolved on 10% SDS-PAGE gel containing 0.1% gelatin under non-denaturizing conditions at 100 V for 2 hours. After electrophoresis, the gel was washed with 2.5% Triton X-100 twice for 40 min. each, and followed by Milli-Q water twice for 20 min. each at room temperature. The gel was soaked with reaction buffer (50 mM Tris-HCl, 5 mM CaCl_2_, 0.02% Brij-35, pH 7.6) for 42 hours at 37°C, stained with 0.25% (w/v) Coomassie brilliant blue G250 in 30% methanol and 10% acetic acid for 3 hours, and destained in methanol-acetic acid-water (30∶10∶70, v/v/v) until the background was homogeneous blue. Areas of protease activity were detected as clear bands against the blue-stained gelatin background.

### Immunofluorescence staining

Transfected MDA-MB-231 cells were labeled using a Cellular NF-κB Translocation Kit (Beyotime, Jiangsu,China) according to the manufacturer's instructions. Briefly, cells were fixed, blocked with the blocking buffer for one hour, and incubated with rabbit anti-human p65 polyclonal antibody for one hour. After washing, the cells were incubated with Cy3-labeled goat anti-rabbit IgG for one hour at room temperature and then stained with DAPI for 5 minutes. The p65 protein (red) and nuclei (blue) were examined through an inverted florescence microscopy (Nikon, TE-2000U, Japan).

### Western blotting assay

The transfected MDA-MB-231 cells were washed twice with ice-cold PBS and then lysed with cell lysis buffer (50 mM NaF, 10 mM Na_2_P_2_O_7_, 2% SDS, 1 mM PMSF). The lysates were collected by scraping from the plates, and then centrifuged at 12000 rpm for 5 min at 4°C. Nuclear and cytoplasmic proteins of MDA-MB-231 cells were extracted by nuclear and cytoplasmic protein extraction kit according to the manufacturer's instructions (Beyotime, Jiangsu, China). The protein concentration was determined by bicinchoninic acid (BCA) assay. Ten µg of lysate was resolved on a 15% of SDS-polyacrylamide gel for electrophoresis (SDS-PAGE) and then transferred to polyvinylidene difluoride (PVDF) membranes. Membranes were blocked at room temperature for 1 hour in tris-buffered saline plus Tween-20 (TBST) (10 mM Tris, 150 mM NaCl, 0.1% Tween-20, pH 7.6) containing 5% nonfat dried milk. Membranes were then incubated with one of the following primary antibodies overnight at 4°C: anti-Hes-1 (1∶1000) (GeneTex, USA), anti-NICD(1∶1000)(Abcam, USA), anti-Bcl-xL (1∶200), anti-Survivin (1∶200), anti-cyclin D1 (1∶200), anti-human p65 (1∶1000), rabbit anti-human IκB (1∶1000), or anti-β-actin (1∶1000) (Boster, Wuhan, China), respectively in TBST containing 1% milk. Membranes were washed three times with TBST containing 1% milk and incubated with appropriate horseradish peroxidase-conjugated secondary antibodies at 1: 2,000-10,000 dilution at room temperature for 2 hours. Membranes were washed three times with TBST and immunoreactive signals were detected by Western Blotting Luminol Reagent (Beyotime, Jiangsu, China). Band densities were then quantified by densitometry.

### Preparation of nuclear extract and Electrophoretic mobility shift assay (EMSA)

MDA-MB-231 cells were transfected as described above. Nuclear extracts were prepared using nuclear and cytoplasmic protein extraction kit (Beyotime) and quantified by Bradford protein assay kit (Beyotime). To perform EMSA, five µg of nuclear extract was incubated with biotin-labeled NF-κB oligonucleotides (Pierce Biotechnology) in a 20 µl reaction containing 1x binding buffer for 20 min at 25°C. The DNA-protein complex was separated from free oligonucleotide on a 4% native polyacrylamide gel using buffer containing 50 mM Tris, 200 mM glycine (pH 8.5), and 1 mM EDTA. Signals were detected by enhanced chemoluminscent assay kit (Beyotime).

### Dual-luciferase reporter assay

For measurement of reporter activity, 3×κB-luciferase reporter plasmid and pRL-TK were co-transfected into MDA-MB-231 cells. Transfected cells were harvested at 48 h after transfection. Luciferase activity was determined using a dual luciferase reporter assay system (Beyotime) according to the manufacture's instructions, detected by a Fluoroskan Ascent FL (Thermo). The relative luciferase activities were normalized for *Renilla* luciferase activity. All conditions were tested in triplicate wells.

### Data presentation and statistical analysis

Results were analyzed using GraphPad Prism Software version 6.0 (GraphPad Software Inc., San Diego, CA) and presented as means ± standard deviation (SD). Statistical analysis was performed using one-way ANOVA. *P*<0.05 was considered statistically significant.

## Results

### Notch-1 regulates proliferation, cell cycle and apoptosis of MDA-MB-231 cells

To determine the effect of Notch-1 signaling on human breast cancer, human breast cancer cell line, MDA-MB-231, was employed as a model system to simulate gain of functions by forced expression of a plasmid encoding human Notch-1 intracellular domain (NICD) or loss of functions by knockdown its expression with Notch-1 shRNA respectively. As shown in Figure 1A, forced expression of NICD up-regulated Notch-1 gene expression 5-fold compared to vector transfected cells, and overexpression of a plasmid encoding Notch-1 shRNA abolished the Notch-1 expression compared to Scrambled shRNA transfected cells, which were further confirmed by Western blot (figure 1B). Overexpression of NICD significantly promoted, whereas knockdown Notch-1 expression significantly inhibited, the proliferation of MDA-MB-231 cells (Figure 2A). In consistent with cell proliferation assay, forced expression of NICD significantly increased, whereas knockdown Notch-1 expression significantly decreased, the colony-forming capability of MDA-MB-231 cell (Figure 2B). We next assessed the anchorage-independent growth that has been shown to correlate well with tumorigenicity *in vivo* [35]. As shown in Figure 2C, overexpression of NICD significantly increased, whereas knockdown the expression of Notch-1 significantly decreased, the number of colonies of MDA-MB-231 cells in soft agar assay.

**Figure 1:** NICD expression assay. The NICD expression was detected by quantitative real-time-PCR assay (**A**) and Western blotting (**B**). ^*^ *P*<0.05 relative to vector and ^#^ *P*<0.01 relative to NICD.

**Figure 2:** Notch-1 promotes MDA-MB-231 cell proliferation. (**A**) MDA-MB-231 cells were seeded in a 96-well plate and transfected with pcDNA3.1(+) (vector), NICD, scrambled shRNA and Notch-1 shRNA. Cell proliferation was assessed by CCK-8 assay after transfection for 48 h. The absorbance values of samples were recorded by a microplate reader at 450 nm. Experimental data were normalized to the control. (**B**) Colony formation assay with transfected MDA-MB-231 cells treated with vector, NICD, scrambled shRNA or Notch-1 shRNA. Cells (4×10^3^) were seeded in 35-mm dishes and continued to culture for 8 days, then the cells were stained with crystal violet. The quantitative colony formation was measured the absorbance at 450 nm. (**C**) The anchorage-independent growth *in vitro*. Transfected cells (3×10^3^) were seeded in 0.3% agarose and incubated for 24 days. Colonies were photographed under a microscope (×40 original magnification). The colony numbers were quantified by clone counting from five microscopic fields for each sample (magnification 10×). Experimental data were normalized to the control. All the results represent the mean ± standard deviation of three independent experiments. ^*^ *P*<0.05 relative to vector and ^#^ *P*<0.01 relative to NICD.

To explore the possible mechanisms of the increased cell proliferation effect of Notch-1 signaling pathway, we performed Calcein-AM/PI co-staining. Forced expression of NICD significantly decreased, whereas knockdown the Notch-1 expression significantly increased, the number of apoptotic cells (PI-positive cells, red) (Figure 3A). To further study the roles of Notch-1 in apoptosis, the transfected cells were stained with Annexin V/PI double-staining and analyzed by flow cytometry. Overexpression of NICD decreased the percentage of apoptotic cells to 0.175% in contrast to 2.52% in vector control, whereas knockdown the Notch-1 expression increased the percentage of apoptotic cells to 14.8% from 4.86% in scrambled shRNA control (Figure 3B). All these results suggested that the activation of Notch-1 signaling pathway protects cells from apoptosis.

**Figure 3:** Notch-1 inhibits MDA-MB-231 cell apoptosis. Cell apoptosis was detected by inverted fluorescence microscope after calcein-AM/PI double staining (**A**) and by flow cytometry using Annexin V-Cy5/PI double staining (**B**) after transfection 72 h, respectively. (*n* = 3)

To investigate whether Notch-1 signaling affects cell cycle distribution, cell cycles were evaluated by flow cytometry. Compared to vector control, overexpression of NICD led to a 14% increase of cells in S phase with a concomitant reduction of cells in both G0/G1 and G2/M phases (Figure 4). Knockdown of Notch-1 resulted in a 10% reduction of cells in S phase and a significant G_0_/G_1_ arrest (Figure 4). Taken together, activation of Notch-1 signaling pathway increases the capacity of anchorage-independent growth and leads to increased proliferation of MDA-MB-231 cells that may come from inhibition of apoptosis and shifting of cell cycle to S phase.

**Figure 4:** Analysis of cell cycle. The cell cycle profiles were determined by flow cytometry using PI staining 72-transfection. (*n* = 3)

### Activation of Notch-1 signaling facilitates adhesion, invasion and motility of MDA-MB-231 cells

To determine the effects of Notch-1 signaling on the malignant features of MDA-MB-231 cells, the adhesion and migration on a modified Millicell cell culture insert were studied. The results showed ectopic expression of NICD significantly increased, whereas knockdown the expression of Notch-1 significantly decreased, the number of adherent cells (Figure 5, p<0.05) and the ability of directional migration (figure 6, p<0.05) when compared to their corresponding controls. We next evaluated the cell mobility and cell scattering of MDA-MB-231 cells using wound-healing assay. Overexpression of NICD significantly accelerated the closure of the wound gap after 24 h (Figure 7, p<0.05). In contrast, knockdown of Notch-1 exhibited limited wound closure activity even after 48 hours (figure 7, p<0.05). These results indicated that the activation of Notch-1 signaling pathway contributes to the increased adhesion, invasion and motility of MDA-MB-231 cells.

**Figure 5:** Notch-1 promotes MDA-MB-231 cell adhesion. (**A**) and (**B**) are the representative images of MDA-MB-231 cells adhesion (labeled in purple) and the statistical data of adhered cell numbers in various conditions, respectively. MDA-MB-231 cells were cultured in Matrigel-coated 24-well plates for 2 h when 48 h post-transfection. The adhered cells were stained with crystal violet, and quantified by cell counting from more than seven microscopic fields using magnification of 20×. ^*^ *P*<0.01 NICD *vs*. vector; ^#^ *P*<0.05 Notch-1 shRNA *vs*. NICD.

**Figure 6:** Evaluation of Notch-1 on MDA-MB-231 cell invasion. (**A**) The cells were transiently transfected for 24 h, then seeded into the Matrigel-coated inner sides of Millicell cell culture inserts. The cells were fixed and stained with crystal violet after 24 h culture, and observed under microscope and photographed (objective 20×). (**B**) The cells invaded into the outer sides of the inserts were counted at five randomly selected fields and represented as mean ± SD. ^*^ *P*<0.05 NICD *vs*. control or vector; ^#^ *P*<0.05 Notch-1 shRNA *vs*. NICD.

**Figure 7:** Evaluation of Notch-1 on cell motility in MDA-MB-231 cells by wound healing assay. (**A**) The cells were transiently transfected for 24 h and then scratched with a pipette tip, and cultured with serum-free media for 24 h or 48 h. The relative wound closure was observed under microscope and photographed (objective 4×). (**B**) Quantification of relative closure of the scratch would was determined via calculating the marked area at nine randomly selected fields by Image J software (NIH, USA), and the data were represented as mean ± SD. ^*^ *P*<0.05 and ^**^ *P*<0.01 relative to control or vector at 48 h.

### Activation of Notch-1 signaling up-regulates MMP-2/9 and VEGF

Accumulating evidence indicates that tumor progression is accompanied with increasing levels of cytokines, chemokines, and MMPs [25], [36]. Recently, increased levels of MMP-2, MMP-9, and VEGF have been reported in breast cancer and levels of which in circulation have been suggested as markers for metastasis [26], [37]. Therefore, we were interested to know whether activation of Notch-1 signaling has any effects on MMP-2, MMP-9 and VEGF. As shown in Figure 8A, ectopic expression of NICD significantly up-regulated (p<0.05), whereas knockdown Notch-1 expression significantly down-regulated (p<0.05), the expression of MMP-2, MMP-9 and VEGF as evaluated by real time-PCR. Consistent with the direct correlation between Notch-1 and MMP-9 gene expression, over-expression of NICD resulted in significantly increased (p<0.05), whereas knockdown Notch-1 expression led to significantly decreased (p<0.05), MMP-9 activity as evaluated by gelatin zymography (Figure 8B). Collectively, these data suggest that activation of Notch-1 signaling up-regulates gene expression of MMP-2, MMP-9 and VEGF, and enzymatic activity of MMP-9.

**Figure 8:** Analysis of Notch-1 on VEGF, MMP-2/9 expression and the activity of MMP-9 in MDA-MB-231 cells. (**A**) Notch-1 signaling regulates VEGF, MMP-2, and MMP-9 mRNA expression of MDA-MB-231 cells by quantitative real-time-PCR assay. (**B**) Zymographic analysis of active MMP-9 expression in non-transfected and transfected MDA-MB-231 cells and quantitatively represented as their gray values. ^*^ *P*<0.05 NICD *vs*. vector; ^#^ *P*<0.01 Notch-1 shRNA *vs*. NICD.

### Activation of Notch-1 signaling induces NF-κB activation

It is well accepted that inflammation, especially chronic inflammation, leads to tumor. As a master regulator of inflammation, NF-κB has been implicated in the onset of most cancers [24]. Hence, we next elucidate whether activation of Notch-1 signaling leads to the activation of NF-κB activation in our MDA-MB-231 model system. As shown in Figures 9A and B, p65 was predominantly localized in the cytosol in control or vector-transfected cells compared to cells overexpressing NICD where p65 was localized mainly in the nucleus, and knockdown Notch-1 expression caused sequestration of p65 in the cytosol compared to cells transfected with scrambled shRNA. Consistent with the increased nuclear translocation of p65 in cells over-expressing NICD, we observed a significant degradation of IκBα that, at resting condition, binds to NF-κB complex and prevents its nuclear translocation (Figure 9C). Moreover, whether Notch-1 signaling had effect on the transcriptional activity of NF-κB promoter is still unknown. To examine this, we co-transfected NF-κB-luc promoter with NICD or Notch-1 shRNA and measured their transcriptional activity. We observed near three-fold upregulation of the promoter in the NICD over-expression cells relative to the vector or scrambled shRNA (Figure 9D). Taken together, Notch-1 signaling could induce NF-κB activation.

**Figure 9:** Notch-1 signaling enhances NF-κB activation and IκBα degradation. (**A**) Cellular distribution of the NF-κB subunit p65 (red) in MDA-MB-231 cells was detected by immunofluorescence staining. The nuclei were stained with DAPI (blue). (**B**) and (**C**) Cells were lysed with lysis buffer. The levels of p65 in total protein, cytosolic extract and nuclear extract (**B**), and IκBα degradation (**C**), were detected by Western blotting. (**D**) NF-κB transcription activity assay by luciferase reporter analysis. The relative luciferase values were calculated by dual luciferase assays. Values shown are averages of at least three separate experiments.

We have shown that activation of Notch-1 signaling caused nuclear translocation of p65 and up-regulated the expression of several NF-κB target genes. To explore the potential mechanisms of Notch-1-mediated up-regulation of NF-κB target genes, the activity of NF-κB was analyzed by EMSA. As shown in Figure 10, overexpression of NICD significantly increased, whereas knockdown Notch-1 expression significantly decreased, the specific DNA-protein complex. These results suggest that Notch-1-mediated growth promoting effects are likely through targeting the promoter of NF-κB target genes.

**Figure 10:** Notch-1 signaling enhances the NF-κB binding activity. EMSA analysis was done for MDA-MB-231 cells. Nuclear extracts were prepared from control and transfected cells and subjected analysis for NF-κB DNA-binding activity as measured by EMSA. Free probe was used as negative control (NC) and the 50 ng/ml tumor necrosis factor-α (TNF-α) stimulated THP-1 cells for 45 min was used as positive control (PC). 100-fold molar excess of unlabeled NF-κB probes were added to untreated cells extracts as competitor control (CC).

### Activation of Notch-1 signaling up-regulates expression of NF-κB target genes

Our data have shown that activation of Notch-1 signaling increased the nuclear localization of NF-κB by immunocytochemistry, Western blotting, and EMSA. To further confirm the activation of NF-κB by increased Notch-1 activity, we analyzed the expression of several genes downstream of NF-κB by Western blot. As expected, overexpression of NICD significantly increased the expression of Hes-1, a Notch-1 signaling molecule, and several NF-κB target genes including Cyclin D1, Bcl-xL and Survivin. In contrast, knockdown Notch-1 expression significantly decreased the expression of those genes (Figure 11). These findings suggest that overexpression of NICD activates Notch-1 signaling and that the growth promoting effects of Notch-1 signaling is likely mediated by NF-κB signaling pathway.

**Figure 11:** Effect of Notch-1 signaling on the expression of Hes-1, cyclin D1, Bcl-xL, and survivin. The expression of Hes-1, cyclin D1, Bcl-xL, and survivin protein was detected by western blotting analysis. The β-actin was used as a loading control.

## Discussion

Notch signaling plays important roles in maintaining the balance between cell proliferation, differentiation, and apoptosis. It has been reported that the Notch gene is abnormally activated in many human malignancies [14], [38], [39]. Therefore, we firstly investigated the effects of Notch-1 signaling on the proliferation of human breast cancer cells. In our study, Notch-1 signaling activation by NICD transfection elicited a dramatic enhancing effect on the growth of MDA-MB-231 cells, as demonstrated by CCK-8 assay and clonogenic assay (Figure 2). However, we observed that knockdown of Notch-1 expression significantly inhibited cell proliferation and colony formation. In addition, down-regulation of Notch-1 caused cell cycle arrest in G0/G1 phase but promoted the apoptosis *in vitro*. Collectively, these data suggested that cell growth enhancement by Notch-1 signaling pathway activation is partly attributed to an inhibition in cell apoptosis and increase in S phase (Figures 3 and 4). It also demonstrated that Notch-1 was a critical regulator of the development of human breast cancer. To further verify the mechanism of Notch-1 promoting cell growth, it was found that Notch-1 pathway activation could up-regulate the expression of cyclin D1, survivin and Bcl-xL, while the down-regulation of Notch-1 leaded to low expression of cyclin D1, survivin and Bcl-xL (Figure 11), suggesting that Notch-1 knockdown arrested cell cycle at G0/G1 might be cyclin D1 dependent, and the inhibition of cell apoptosis might be related to elevated expression of both survivin and Bcl-xL.

Cell adhesion, invasion and motility are fundamental processes required for metastatic spread of a primary tumor, which are pivotal steps in the intricate process of tumor metastasis [40]. A high expression level of Notch-1 has also been found to play an important role in the metastasis in many cell types [13], [27], [41]. To determine the role of Notch-1 signaling in the metastasis behaviors, we then examined the effect of Notch-1 signaling on cell adhesion, invasion and motility. It was found that the adhesion, invasion and motility of MDA-MB-231 cells transfected with NICD were significantly increased (Figures 5, 6 and 7). In parallel, this finding was also supported by Notch-1 knockdown in the Notch-1 shRNA transfected cells, which remarkably inhibited cell adhesion, invasion and motility. These data implied that the cells with Notch-1 signal activation had a greater invasive potential. However, the precise mechanism of Notch-1 signaling for promoting cancer cell metastasis remains unclear. It is well accepted that many important molecules, such as MMP-2, MMP-9, VEGF, are involved in tumor cell invasion and metastasis [36], [42]. Hence, we further explored the effects of Notch-1 signaling activation by NICD transfection or down-regulation of Notch-1 by Notch-1 shRNA transfection on expression and activity of the above-mentioned molecules. We found that Notch-1 signaling enhanced the expression of MMP-2, MMP-9 and VEGF as well as the activity of MMP-9 (Figure 8), which was well consistent with the phenotype of adhesion, invasion and motility of MDA-MB-231 cells. It suggested that the Notch-1 signaling-induced cell invasive growth was partly due to the up-regulation of MMP-2, MMP-9 and VEGF, and the down-regulation of Notch-1is likely to have beneficial effects for the prevention of breast cancer.

Although several studies have shown the functional significance of Notch signaling, the Notch-1 pathway in breast cancer remains to be poorly elucidated [11], [17]. Therefore, we further investigated the mechanisms of Notch-1 signaling in the proliferation and migration of MDA-MB-231 cells. It has been reported that NF-κB controls the expression of the cytoplasmic inhibitor of apoptosis protein, and then blocks the activation of caspases and Bcl-xL, which is an anti-apoptotic gene of the Bcl-2 family. NF-κB is also a pleiotropic transcription factor that is associated with metastatic phenotype and regulates the expression of a variety of important genes in some cellular responses, including the MMP-2, MMP-9 and VEGF, which are associated with cell migration and invasion [27], [37]. Recently, the cross-talking of various signal pathways has been received attention. In this study, we found that down-regulation of Notch-1 by Notch-1 shRNA transfection significantly decreased p65 nuclear translocation and NF-κB DNA-binding activity in MDA-MB-231 cells. However, Notch-1 pathway activation by NICD transfection strongly induced NF-κB activation and NF-κB DNA binding activity (Figures 9 and 10). These data suggested that Notch-1 activation maintains NF-κB activity. It was also demonstrated that Notch-1 signaling activation could lead to NF-κB activation, while deactivation of Notch-1 could inhibit NF-κB activity. Taken together, these results demonstrated that Notch-1 signaling could promote breast cancer cell invasion and motility, partly due to the activation of NF-κB and its downstream target genes such as MMP-2, MMP-9 and VEGF.

In conclusion, in this paper, we presented experimental evidence which supported that Notch-1 signaling promoted invasive growth of MDA-MB-231 cells, including adhesion, invasion and motility through activating NF-κB pathway, and the expression level of Notch-1 was also associated with the growth and migration of breast cancer MDA-MB-231 cells. Down regulation of Notch-1 could be an effective approach for the deactivation of NF-κB and its target genes, such as MMP-2, MMP-9, and VEGF, which then inhibits cell migration and invasion. Moreover, our data also provided mechanistic information that the down regulation of Notch-1 arrested cell cycle and promoted cell apoptosis, which were related to the gene expression decrease of cyclin D1, survivin, and Bcl-xL. Based on our results, we proposed a hypothetical pathway (Figure 12) by which Notch-1 signaling regulates cell growth, migration and invasion, although further studies for the specific mechanisms are still needed. We believe that Notch-1 and NF-κB are intimate partners in the process of tumor aggressiveness, and thus targeted deactivation of these pathways might provide a new therapeutic strategy for the treatment of breast cancer in the future.

**Figure 12:** Schematic illustration of Notch-1 signal pathway to regulate gene expression. This model summarizes our findings that Notch-1 activation promotes the malignant features of human breast cancer MDA-MB-231 cells via cross-talking the NF-κB signal pathway.
